# Comparison of Febuxostat and Allopurinol in the Treatment of Patients with Chronic Kidney Disease Stage 3∼5 with Hyperuricemia

**DOI:** 10.1155/2022/1177946

**Published:** 2022-10-11

**Authors:** Zhimin Liao, Lei Xu, Bo Wan, Liping Wang, Chengzhi Zhao, Gang Wu, Rui Xie

**Affiliations:** ^1^Department of Nephrology, The Second People's Hospital of Liangshan Yi Autonomous Prefecture, Xichang, Sichuan 615000, China; ^2^The Second People's Hospital of Liangshan Yi Autonomous Prefecture, Xichang, Sichuan 615000, China

## Abstract

**Objective:**

To compare the efficacy of febuxostat and allopurinol in the treatment of chronic kidney disease (CKD) at stages 3∼5 with hyperuricemia.

**Methods:**

A total of 100 patients with stage 3 to 5 CKD with hyperuricemia in our hospital from July 2018 to December 2019 were selected and divided into the control group (*n* = 50) and the experimental group (*n* = 50) according to the random number expression method, the control group on the basis of conventional treatment with allopurinol treatment, the experimental group based on conventional treatment using the febuxostat be treatment. The clinical efficacy, incidence of adverse reactions, and renal function indexes, blood urea nitrogen (BUN), serum creatinine (Scr), serum sodium (Na), serum potassium (K), and serum uric acid (UA) before and after treatment were compared between the two groups.

**Results:**

The total effective rate of the experimental group and the control group was 82.00% and 78.00%, respectively, with little difference (*P* > 0.05); compared with before treatment, BUN, Scr, and UA of the two groups were decreased (*P* < 0.05); and the degree of decline in the experimental group was significantly greater than that in the control group (*P* < 0.05); the incidence of adverse reactions in the control group was 22.00%, which was significantly higher than that in the experimental group (10.00%) (*P* < 0.05).

**Conclusion:**

Compared with allopurinol, febuxostat can improve renal function, reduce UA levels, and reduce the occurrence of complications, with high safety, which is worthy of further clinical promotion.

## 1. Introduction

Chronic kidney disease (CKD) is a common nephrology disease. It is mainly caused by renal function and renal structural disorders caused by various factors. With the continuous deterioration of the disease, it will lead to the retention of metabolites, water, electrolyte, and acid-base balance disorders in patients. Hyperuricemia is one of the important factors leading to the development of CKD [1, 2]. Studies have shown that hyperuricemia is gradually showing a younger trend, accounting for 10% of the population, and it is very easy to cause heart disease, hypertension, diabetes, hyperlipidemia, and other diseases [3]. In view of the important mechanism of serum uric acid in the pathogenesis of CKD, we can conclude that how to effectively improve CKD and reduce the serum uric acid value is particularly important for patients with CKD stage 3–5 combined with hyperuricemia. The most commonly used uric acid-lowering drugs in clinical practice include febuxostat and allopurinol, but there are few reports on the efficacy of these two drugs in patients with CKD and their differences [4–6]. Therefore, this study selected 100 patients with CKD stages 3–5 with hyperuricemia who were admitted to our hospital from July 2018 to December 2019, and compare the therapeutic effects of febuxostat and allopurinol in the treatment of CKD at stages 3–5, the report is as follows.

## 2. Materials and Methods

### 2.1. Research Objects

This study selected 100 patients with CKD stage 3 to 5 with hyperuricemia who were admitted to our hospital from July 2018 to December 2019 and divided them into the control group (*n* = 50) and the experimental group (*n* = 50) according to the random number expression method. In the experimental group, there were 32 males and 18 females, the age ranged from 33 to 83 years old, and the average age was (63.80 ± 4.21) years old, there were 20 cases in stage 3, 21 cases in stage 4, and 9 cases in stage 5. In the control group, there were 30 males and 20 females, the age ranged from 31 to 85 years old, and the average age was (64.13 ± 5.10) years old, there were 22 cases in stage 3, 21 cases in stage 4, and 7 cases in stage 5. There was no significant difference in the general data such as gender, age, weight, and education level between the two groups (*P* > 0.05), which is comparable. See Table 1 for details. Inclusion criteria were as follows: (1) blood uric acid (UA) >360 *μ*mol/L in females and UA > 420 *μ*mol/L in males; (2) CKD stage 3–5 with hyperuricemia, serum creatinine (Scr) is about 133–442 *μ*mol/L; (3) meet the diagnostic criteria for CKD in the guidelines of the “Kidney Disease Prognosis Quality Initiative” published by the National Kidney Foundation [7]; (4) this study was approved by the Medical Ethics Committee, and patients or their families gave informed consent to the study and signed the informed consent form voluntarily. Exclusion criteria were as follows: (1) combined with malignant tumor; (2) those with severe insufficiency of organs such as the heart, liver, or lung; (3) patients who are allergic to the drugs in this study; (4) those with mental disorders or cognitive impairments; (5) the general information is incomplete or the researcher quits midway.

### 2.2. Treatment Methods

The patients in both groups received conventional treatments such as supplementing *α*-keto acid, correcting water, electrolyte, and acid-base balance, reducing blood pressure, improving anemia symptoms, ensuring a high-quality low-protein, and low-purine diet. Control group: oral 100 mg allopurinol (Guangzhou Bidi Pharmaceutical Co., Ltd., Chinese medicine Zhunzi: S14202000669, specification: 100 mg) once a day; experimental group: oral 40 mg febuxostat (Jiangsu Wanbang Biochemical Pharmaceutical Co., Ltd., specification: 40 mg) 1 time/d.

### 2.3. Observation Indicators

The clinical efficacy, the incidence of adverse reactions, renal function indexes blood urea nitrogen (BUN), serum creatinine (Scr), serum sodium (Na), serum potassium (K), and UA before and after treatment were compared between the two groups.

### 2.4. Detection Method

(1) Clinical curative effect: Significant effect: Scr decreased by more than 50% compared with that before treatment, UA decreased by more than 20% compared with that before treatment, and the clinical symptoms of patients disappeared; valid: Scr decreased by more than 20%–50% and UA decreased by more than 10%–20% compared with that before treatment, and the clinical symptoms of patients were improved; invalid: Scr and UA increased, and the patient's clinical symptoms were not relieved or even aggravated. Total effective rate = (Significant effective cases + Valid cases)/Total cases × 100%. (2) Renal function index: 5 ml of cubital venous blood was collected from the patient in the morning and on an empty stomach, centrifuged at 4°C, and sent to the laboratory. PUZS-300 automatic biochemical analyzer (Shanghai Huanxi Medical Instrument Co., Ltd.) was used to detect the Scr, Na, BUN, and K levels. of the patient before and after treatment. (3) UA: 5 ml of venous blood was drawn, placed in an EDTA anticoagulant tube, centrifuged at 3000 r/min for 10 min, and the plasma was separated. The supernatant was collected, and the UA level was detected by capillary electrophoresis. The kit was from Shanghai Xuanhao Technology Development Co., Ltd. company. According to the instructions of the kit and the instrument, it will be strictly carried out by special personnel.

### 2.5. Statistical Methods

All data were processed by SPSS 23.0 statistical software package, measurement data were expressed as mean ± standard deviation (Mean ± SD), and a *t*-test was used; the pass rate/composition ratio of count data was described by the *χ*^2^ test, and *P* < 0.05 was considered statistically significant for differences.

## 3. Results

### 3.1. Comparison of Clinical Efficacy between the Two Groups

The total effective rates of the experimental group and the control group were 82.00% and 76.00%, respectively, and the difference was not statistically significant (*P* > 0.05), as shown in Table 2.

### 3.2. Comparison of UA and Renal Function Indexes between the Two Groups before and after Treatment

Compared with before treatment, BUN, Scr, and UA in both groups decreased after treatment (*P* < 0.05); and the degree of decrease in the experimental group was significantly greater than that in the control group (*P* < 0.05). As shown in Table 3.

### 3.3. Comparison of the Incidence of Adverse Reactions between the Two Groups after Treatment

The incidence of adverse reactions in the control group was 22.00%, which was significantly higher than that in the experimental group (10.00%) (*P* < 0.05). As shown in Table 4.

## 4. Discussion

As the kidney is an important organ for the excretion of uric acid, when the proximal convoluted renal tubule increases the reabsorption of uric acid and the glomerular filtration rate is reduced, it can lead to secondary hyperuricemia in patients with chronic renal failure. In addition, the metabolic disorder caused by chronic renal disease is also one of the important reasons for hyperuricemia [8, 9]. Uric acid accumulation in the kidney can activate renin-angiotensin inhibit epithelial-mesenchymal transdifferentiation, nitric oxide synthase-aldosterone system, trigger an inflammatory response, oxidative stress, etc., and eventually lead to tubulointerstitial damage and renal vascular disease, which is also an important reason for the exacerbation of CKD [10]. Studies have shown that renal dysfunction and hyperuricemia have far more influence on patients with CKD than that of proteinuria, and they are the main factors affecting the development of patients' conditions. [11]. Therefore, how to effectively control hyperuricemia is an important part of the treatment of CKD. At present, the treatment of CKD with hyperuricemia is mainly aimed at promoting uric acid excretion and inhibiting uric acid synthesis. Allopurinol is one of the drugs commonly used in the clinical treatment of hyperuricemia. Its main mechanism is to reduce uric acid synthesis. Inhibit the metabolism of xanthine and hypoxanthine. However, relevant data show that the use of allopurinol in the treatment of CKD with hyperuricemia has not achieved an ideal therapeutic effect, and the incidence of adverse reactions is high [12, 13]. In this study, the incidence of adverse reactions in the control group was 22.00%, which was significantly higher than that in the experimental group (10.00%) (*P* < 0.05), which was in line with the aforementioned data. This shows that the incidence of adverse reactions in patients with CKD and hyperuricemia treated with allopurinol is significantly higher than that of febuxostat.

Febuxostat was launched in China in 2013 [14], but there is no systematic report on the safety, experience, and efficacy of febuxostat in the field of kidney disease. Febuxostat mainly inhibits uric acid synthesis by selectively inhibiting xanthine oxidase. It is a novel uric acid-lowering drug that inhibits oxidative xanthoxylum and reductase from being affected by purinase such as pyrimidine metabolism. Therefore, febuxostat can effectively reduce drug damage to the body, accelerate the excretion of uric acid, improve the reduction efficiency of uric acid, is not affected by the redox state of enzymes, and ensure that no dose resistance is generated during the treatment [15–17]. At the same time, it can be converted into inactive products by the metabolic function of the liver, and finally eliminated from the body. Compared with allopurinol or other uric acid-lowering drugs currently in clinical use, febuxostat has a more significant treatment effect and has less impact on patients' renal function. In some developed countries, febuxostat has been used for chronic hyperuricemia in patients with a history of gouty joints and gout and has achieved good results [6, 18]. In this study, BUN, Scr, and UA in the two groups decreased after treatment (*P* < 0.05); and the degree of decrease in the experimental group was significantly greater than that in the control group (*P* < 0.05), indicating that febuxostat can effectively reduce the effect of hyperuricemia on renal function of patients. To analyze the reason, febuxostat can increase glomerular filtration rate, improve the renal function of patients, and promote the recovery of renal function, so as to avoid the rise of intrarenal pressure of surviving nephrons, leading to the hypertrophy of arteriole wall, and thus, reducing the renal impairment and urinary protein precipitation. [19].

In conclusion, compared with allopurinol, febuxostat can improve renal function, reduce UA level, and reduce the occurrence of complications, with high safety, which is worthy of further clinical promotion. However, due to the limitation of the small sample size and short observation time in this study, it is necessary to increase the sample size and extend the observation time in subsequent studies for further discussion.

## Figures and Tables

**Table 1:** Comparison of general information of patients (*n*%, (±*S*)).

Group	*N*	Age (year)	Gender		Weight (kg)	Education level			
			Male	Female		College and above	High school	Junior high school	Elementary school and below
Experimental group	50	63.80 ± 4.21	32	18	44.17 ± 3.12	12	16	9	13
Control group	50	64.13 ± 5.10	30	20	45.34 ± 3.54	15	12	10	13
*t* value	—	1.547	0.524		2.356	1.302			
*P* value	—	0.074	0.492		0.065	0.954			

**Table 2:** Comparison of clinical efficacy between the two groups [*n* (%)].

Group	*n*	Significant effect	Valid	Invalid	Total efficiency
Control group	50	15	24	11	39 (78.00)
Experimental group	50	16	25	9	41 (82.00)
*t* value	—	—	—	—	3.827
*P* value	—	—	—	—	> 0.05

**Table 3:** Comparison of UA and renal function indexes between the two groups before and after treatment (±S).

Group	*N*		BUN (mmol/L)	Scr (mmol/L)	Na (mmol/L)	K (mmol/L)	UA (*μ*mol/L)
Control group	50	Before treatment	17.24 ± 5.05	326.32 ± 56.24	127.21 ± 12.47	3.36 ± 0.92	503.64 ± 50.31
		After treatment	12.44 ± 5.15^a^	275.15 ± 41.62^a^	130.35 ± 11.42	3.41 ± 7.39	446.35 ± 42.35^a^
Experimental group	50	Before treatment	18.32 ± 4.24	326.23 ± 57.52	128.75 ± 11.24	3.38 ± 1.23	498.36 ± 50.25
		After treatment	10.24 ± 4.11^ab^	243.25 ± 41.25^ab^	131.24 ± 15.67	3.14 ± 0.32	361.58 ± 28.67^ab^

*Note.* Compared with before treatment, ^a^*P* < 0.05; compared with the control group after treatment, ^b^*P* < 0.05.

**Table 4:** Comparison of the incidence of adverse reactions between the two groups after treatment [*n* (%)].

Group	*n*	Rash	Abnormal liver function	Gastrointestinal functional response	Allergic vasculitis	The incidence of adverse reactions
Control group	50	2	4	3	2	11 (22.00)
Experimental group	50	1	1	2	1	5 (10.00)
*t* value	—	—	—	—	—	5.31
*P* value	—	—	—	—	—	< 0.05

## Data Availability

The data can be obtained from the corresponding author upon reasonable request.
